# Teaching Mode of Basic Piano Course in Colleges Based on Students' Application Ability under FC Environment

This article has been retracted.

**DOI:** 10.1155/2022/4710520

**Published:** 2022-09-14

**Authors:** Lin Li

**Affiliations:** Anshan Normal University, Liaoning, Anshan 114000, China

## Abstract

With the popularization of piano education, various schools are constantly carrying out reforms in order to cultivate piano application-oriented talents. While accelerating the creation of a perfect piano teaching model, they are also striving to adapt to the trend of the times. The basic education of piano in colleges and universities is a training activity for musicians, and this education method directly affects the professional quality of music of students. How to learn basic piano is very worthy of attention. Basic piano education is a thorough training of piano in conventional colleges, which can improve practical strength and the capacity to apply music broadly. The main purpose of teaching the fundamentals of piano is to develop students' visual acuity and help them comprehend and apply the principles of aesthetics. The teaching approach for beginning piano classes at various schools is still in its infancy and is deficient in every way. This essay examines the “flipped classroom (FC)” teaching approach used to offer beginner piano lessons in a number of schools. This study proposes the specific process of the “FC” teaching mode and explores the implementation impact of particular scenarios, specifically in light of the features of the training mode of applied abilities. Through inquiry and research, it has been determined that students who get FC instruction have greater employment rates than those who receive traditional instruction, with an average rise of 14.2 percent and a maximum increase of 17 percent. Based on the students' application skills, it demonstrates that the FC teaching technique is generally successful for the teaching method of basic piano courses in colleges and universities.

## 1. Introduction

Nowadays, music education is an important part of quality education in colleges and universities, and it must adapt to the rapid development of social economy. Its development direction has also attracted more and more attention. Music may promote personal cultivation and quality, as well as cultivate people's sentiments and alter their temperaments. For music majors in comprehensive at several schools, the piano foundation course is a prerequisite. This course is crucial because it gives students the opportunity to master a new skill and broaden their scope of practical application. However, when it comes to the training goals of piano instruction in comprehensive colleges and universities, schools must foster their students' aptitude for application. Piano performance, which is primarily to develop performative talents rather than application ability, is extremely different from this. As the times demand, more and more creative teaching methods arise with the development and promotion of various teaching methods in schools. The study of the FC teaching mode has elevated to a top priority for the basic piano course teaching mode in many schools depending on students' application abilities.

The ability to improvise piano accompaniment is especially crucial for college students to acquire in order to strengthen their piano application skills, according to research and practice. Cook thought that pupils in basic piano classes typically had issues with their advanced age, weak piano foundations, and hard fingers, which created significant teaching challenges [1]. The upgraded FC is utilised for instruction to increase students' all-around competence when teaching Pya's basic piano curriculum in different schools [2]. In order to ensure that pupils have a high level of focus and motivation when learning the material, Aldhafiri and Alshaye encouraged students to actively participate in the teaching process. This increased their drive to learn the piano. It encourages student performance and teamwork while upholding the fundamental stability of fundamental piano lessons [3]. Al-Mofti thought that piano instruction should be properly combined with the features of their individual majors since some students are not professional music students [4]. Frcs found that for vocal music students, the methods of their classes should be used to help students understand piano music and music processing. It starts from the songs adapted from the songs, from the shallow to the deep, polyphonic music, sonatas, etc. When necessary, teachers can ask students to sing the melody of the piano music by themselves [5]. Ma believed that in the basic teaching of piano in various schools, the cultivation of application ability is extremely important [6]. Tabuena proposed that improvisational accompaniment is a compulsory course in the basic course of piano education. In addition to mastering the basic knowledge of piano performance, it is also very important to strengthen the practical training of performance [7]. Therefore, the mastery and application of piano impromptu accompaniment skills is one of the important criteria to measure their future work ability.

The FC is a novel kind of instruction in conventional classroom settings. The unique educational foundation of the present determines the development and effective use of the FC. With the basic piano course taught using the FC teaching method as the research object, Geng and Zhang aimed to examine the course's definition, developmental traits, and fundamental meaning [8]. Yu was dedicated to exposing the distinctions between the traditional piano basic courses taught in colleges and the FC basic courses taught in various schools [9]. From the viewpoints of philosophy and practice, Qing explored the trajectory of the FC teaching mode. For the innovation of the FC teaching method, a localization strategy system is suggested [10]. The internalization of knowledge in the classroom and the completeness of knowledge transfer outside the classroom were both stressed by Bai [11]. On the basis of analyzing the current situation of basic piano course teaching in colleges and universities, Wang applied the FC teaching mode to the teaching of basic piano courses in various schools [12]. Li's research found that “flipped classroom” is a brand-new teaching mode that subverts the traditional teaching process, including teaching and internalizing knowledge, embodying the “student-centered” teaching philosophy [13]. Xiaoru has studied the “flipped classroom” teaching mode in the experimental teaching of basic piano courses in various schools. Especially in view of the characteristics of the training mode of applied talents, he designed the specific process of the “flipped classroom” teaching mode and discussed the implementation of specific cases [14]. Li believed that the core of the FC teaching model is to learn first and then teach. This teaching mode was that after completing all the online materials prescribed by the teacher, students go to the classroom to discuss with the teacher and classmates, which helps to improve classroom interaction and meet the individual needs of students [15]. Combined with the educational goals of various schools, the FC teaching mode is applied to the teaching of basic piano courses in various schools, aiming to improve the effectiveness of the curriculum and students' practical ability.

The advancement of science and technology has had a significant impact on all facets of people's lives, and it also applies to how all facets of life will develop in the future. Education cannot go back to general development because it was the cornerstone of the twentieth century. We can only satisfy the demand for applicable abilities in society by innovating and evolving with the times. The way that education is currently conducted has experienced significant modifications as a result of the use of technology. Following the rise of other new teaching approaches, “FC” has opened up new development options for piano education across a variety of schools. This marks a significant turning point in the development of piano education across the board in educational institutions. Through the approach of data evaluation and analysis, this research explores the current changes in the form of piano teaching in various schools and the teaching manner of FC various schools.

## 2. Teaching Mode of Basic Piano Course in Various Schools Based on Application Ability

### 2.1. Status Quo of Applied Talents and Training Modes

Applied talents refer to talents who, under the guidance of certain scientific principles, combine social interests and apply knowledge in practice and can be directly used in social construction after school education. It can effectively connect school education and social needs [16], as shown in Figure 1.

Application-oriented talents are a subset of specialised talents that can apply professional knowledge and skills to the professional social practice they are involved in. They also possess specific application and comprehensive abilities. Instead of scientific discovery and knowledge generation, applied talents mostly consist of applied knowledge. The need for practical talents in the restructuring of higher education is widespread in society.

### 2.2. The Difference between FC and Traditional Teaching

In the information age, FC is a new kind of teaching strategy. The comprehensive ability of both students and teachers is greatly enhanced by this teaching method, which has a direct positive impact on the conventional teaching approach. This method of instruction is currently in use as well, and Figure 2 illustrates how it differs from the conventional teaching strategy.

The change in learning subject and the emphasis on knowledge teaching, which is embodied in the teaching process, distinguish the FC from the traditional classroom. In the flipped classroom, the emphasis is placed less on “teaching in the classroom” and more on “internalization and absorption after class,” with students serving as the primary source of knowledge acquisition. The FC is intended to liberate educators from repeated knowledge emphasis and conventional resilience learning methods. In order to encourage students to complete the acquisition of knowledge in the classroom, it gives more attention to the analysis of the learning situation of the students and conducts preclass preparations and classroom activities. This gradually strengthens students' capacity for independent learning as well as their capacity for problem-solving and analysis. Traditional educators are weary of constantly reiterating lessons and knowledge points. They take on a leading role in the teaching interaction and must invest a lot of time in the classroom to teach students new material. In this way, it is challenging to finish the necessary teaching tasks, and it is difficult to effectively develop students' all-around abilities.

### 2.3. The FC Teaching Mode in Colleges and Universities Based on the Cultivation of Application Ability

The learning style of college students has advanced to a new level as a result of the quick development of information technology [17]. The FC refers to the reversal of the two stages of knowledge imparting and knowledge internalization in the traditional learning process, where students finish the teaching of preclass knowledge through videos and teaching materials prepared by teachers before class and concentrate on solving problems in class. By receiving timely feedback and evaluation, students can actively summarize and reflect after class, which can better cultivate students' autonomous learning ability and application ability, as shown in Figure 3.

### 2.4. Circular Four-Stage Model of FC

The circular FC is another name for the FC that is frequently used. Experience participation, concept exploration, meaning construction, and display application are the four stages that make up the entire teaching process. Usually starting with participatory learning activities, students complete the exploration of concepts by watching instructional videos, consulting online materials, and participating in online exchanges. Then, they conducted tests, wrote articles to complete meaning construction, and finally presented personalized items in group discussions to complete knowledge application. The flipped classroom structure presented by this model is most in line with the constructivism of the “leader.” The four elements of flipped classroom are “scenario,” “collaboration,” “conversation,” and “meaning construction.” It truly embodies the process of teachers as facilitators to help guide students' learning, as shown in Figure 4.

The teaching philosophy of FC is in line with the learning characteristics of college students, which is why it is preferred by educators and students in a variety of schools. For both students and teachers, the FC teaching mode fosters a generally welcoming and peaceful environment. The discussion and reflection that takes place between students and teachers piques students' interest and makes learning more adaptable and active.

## 3. Application of Text Classification Algorithm in Flipped Classroom Teaching Mode

This paper uses a variety of text classification algorithms to the flipped classroom teaching mode in order to better illustrate the practical effect, with the goal of giving students more effective learning resources for fundamental piano lessons [18].

### 3.1. Bernoulli Naive Bayes Algorithm

For a document *d*, it is represented in the vector form*d* = {*a*_1_*a*_2_, *a*_3_, ⋯*a*_*n*_}, *a*_*i*_ ∈ {0, 1}, where *a*_*i*_ = 1 indicates that the word appears in document *d*; otherwise, it does not appear, and *n* indicates the size of the dictionary; the formula is expressed as

(1) $$\begin{array}{c} c\left(d\right)={amg}_{c\in C}\max j\left(o\right)\overset{n}{\underset{i=1}{\prod }}\left(a_{n}+1\right)+\left(1-a_{n}\right)p, \end{array}$$

where (1 − *a*_*n*_) can represent the conditional probability, which is approximated by frequency count. The calculation formula is

(2) $$\begin{array}{c} \left(1-a_{n}\right)=\frac{m_{\text{in}}}{m_{n}}, \end{array}$$

where *m*_in_ represents the number of documents in class *c* where the word *a*_1_ appears and *m*_*n*_the number of documents belonging to class *c*. Generally, smooth estimation is used, and the specific calculation is shown in the formula:

(3) $$\begin{array}{c} \left(1-a_{n}\right)=\frac{\sum_{0=1}^{n}a_{i}\left(ni,n\right)+1}{\sum_{0=1}^{n}a_{i}\left(ni,n\right)+2} \end{array}$$

*ℓ*(•) is a binary function, which is 1 when the parameters are equal and 0 otherwise, and the calculation formula of the prior probability *p*(*a*)is

(4) $$\begin{array}{c} p\left(a\right)\frac{\sum_{0=1}^{n}\ell \left(n_{i},n\right)}{m} \end{array}$$

### 3.2. AdaBoost Algorithm and Its Optimization

The principle of AdaBoost algorithm is as follows:

1. Input a training set *K* = {(*a*_1_, *b*_1_), (*a*_2_, *b*_2_), ⋯, (*a*_*n*_, *b*_*n*_)} of size *n*, where *b* is the class label of the corresponding instance *a*
2. Initialize the weight of each text in the training set *K*, *w*_1*i*_ = 1/*n*
3. According to the weight vectore *w*_1_, *m* samples are randomly selected from *K* as a new training set new *K*, weight matrix *w*_*n*_ = (*w*_*n*1,_*w*_*n*2_, ⋯, *w*_*n*_*m*)
4. Train the weak classification model *h* on the training set new *K*, and then calculate the weight classification error*q*_*h*_ during the training process

(5) $$\begin{array}{c} q_{h}=M\left(h\left(t_{i}\right)\neq l_{i}\right)=\overset{n}{\underset{n=1}{\sum }}w_{n}p\left(\neq l_{i}\right) \end{array}$$

(5) Calculate the discourse power of the weak classifier *h*

(6) $$\begin{array}{c} a_{h}=\frac{1}{2}pn\frac{1-q_{n}}{q_{n}} \end{array}$$

(6) Update the weight matrix *w*_*n*+1_ = (*w*_*n*+1_, 1, *w*_*n*+1_, 2, ⋯, *w*_*n*+1_, *u*, ⋯, *w*_*n*+1_, *m*); the formula is:

(7) $$\begin{array}{c} w_{n+1},u=\frac{w_{n,u}}{z_{t}}\exp\left(-\alpha_{n}l_{i}h\left(t_{i}\right)\right),u=1,2,\cdots ,n. \end{array}$$

*Z*_*t*_is the normalization factor, the sum of all weights is 1, and the formula is:

(8) $$\begin{array}{c} Z_{t}=\overset{u}{\underset{i=1}{\sum }}w_{n},i\exp\left(-\alpha_{n}l_{i}h\left(t_{i}\right)\right) \end{array}$$

(7) Repeat the above steps to train *K* weak classifiers
(8) The final classifier is obtained as

(9) $$\begin{array}{c} N\left(a\right)=\mathrm{sign}\;\left(\overset{o}{\underset{o=0}{\sum }}\alpha_{o}h_{o}\left(a\right)\right) \end{array}$$

In most cases, when the number of weak classifiers is large enough, the AdaBoost algorithm can show sufficiently superior performance.

### 3.3. Naive Bayes Algorithm

Naive Bayes algorithm is a new classification model based on Bayes' theorem, which is one of the commonly used classification methods in statistics [19]. “Naive”: it is assumed that the contribution of feature items to determining which category the text belongs to is independent of each other; that is, the feature items in the text are independent of each other.

Assume that the text to be classified is *d*_*j*_ = (*a*_1_, *a*_2_, ⋯*a*_*n*_), the category set is*B* = (*b*_1_, *b*_2_, . ⋯ *b*_*m*_), and *a*_1_refers to the weight value of all feature items in the text *d*_*j*_. *n* refers to the total number of all feature items of *d*_*j*_ in the text, and *m* refers to the total number of all categories, so, for text*d*_*j*_ and category *c*_*o*_ can be calculated as follows:

(10) $$\begin{array}{c} A\left(c_{o}\left|d_{j}\right.\right)=\frac{A\left(d_{j}\left|c_{o}\right.\right)A\left(c_{o}\right)}{A\left(d_{j}\right)}, \end{array}$$

where *A*(*c*_*o*_) is the prior probability of category *c*_*o*_ and the calculated value is the ratio of the number of texts in category *c*_*o*_ to the total number of all texts in the training set. Since the *A*(*d*_*j*_) values are the same, the original formula can be simplified to get:

(11) $$\begin{array}{c} A\left(c_{o}\left|d_{j}\right.\right)=A\left(d_{j}\left|c_{o}\right.\right)A\left(C_{o}\right). \end{array}$$

According to the assumption of independence between features, *A*(*d*_*j*_|*c*_*o*_) can be expressed as

(12) $$\begin{array}{c} A\left(d_{j}\left|c_{o}\right.\right)=\overset{n}{\underset{u=1}{\sum }}A\left(w_{uj}\left|c_{o}\right.\right). \end{array}$$

Among them, the value of *A*(*w*_*uj*_|*c*_*o*_) can be calculated as

(13) $$\begin{array}{c} A\left(c_{o}\left|d_{j}\right.\right)=A\left(c_{o}\right)\;\overset{n}{\underset{u=1}{\sum }}A\left(w_{uj}\left|c_{o}\right.\right). \end{array}$$

The advantages of the Naive Bayes algorithm: the algorithm is simple, the execution speed is fast, and the accuracy of the classification results is high. The algorithm's assumption of independence between feature items may lead to inaccurate classification results of the classifier [20].

Given the document *d* to be tested, the MNB model uses the following formula to predict document *d*:

(14) $$\begin{array}{c} c\left(d\right)={amg}_{a\in A}amx{\left[\log_{2}\;A\left(c\right)+\overset{n}{\underset{u=1}{\sum }}s_{u}\;\log\right]}_{2}. \end{array}$$

The prior probability *A*(*c*) can expressed in an algorithmic formula as

(15) $$\begin{array}{c} A\left(c\right)=\frac{\sum_{u=1}^{n}\delta \left(c_{u},c\right)+1}{m+1}. \end{array}$$

The formula for conditional probability is

(16) $$\begin{array}{c} A\left(w_{n}\left|c\right.\right)=\frac{\sum_{u=1}^{n}s_{u}\delta \left(c_{u,}c\right)+1}{\sum_{u=1}^{m}\sum_{u=1}^{n}s_{u}\delta \left(c_{u},c\right)+m-1}. \end{array}$$

After training and testing a classification model has been implemented, evaluating the performance of the classification model is also an important step in the classification process.

The precision rate represents the ratio of the number of samples accurately identified as *C*_*a*_ by the classification model to the total number of texts identified by the classification model as *C*_*a*_ in all categories. It is to measure the accuracy of the classification text system, and the specific calculation method is

(17) $$\begin{array}{c} A=\frac{TB}{TB+FB}. \end{array}$$

The recall rate represents the ratio of the number of samples that the classification model accurately discriminates as category *C*_*a*_ to the total number of samples of all categories *C*_*a*_ in the real situation. It is used to measure the completeness of the classification system, and the specific calculation method is

(18) $$\begin{array}{c} B=\frac{TB}{TB+FQ}. \end{array}$$

The effects of precision and recall are jointly considered, and the comprehensive calculation method is as follows:

(19) $$\begin{array}{c} R_{1}=\frac{2\left(AB\right)}{A+B}. \end{array}$$

Now suppose that there are *m* categories in the category set, the text set calculation formulas are

(20) $$\begin{array}{c} \text{MicAmg}\_A=\frac{\sum_{u=1}^{n}{TB}_{u}}{\sum_{u=1}^{n}\left({TB}_{u}+{FB}_{u}\right)}, \end{array}$$

(21) $$\begin{array}{c} \text{MicAmg}\_B=\frac{\sum_{u=1}^{n}{TB}_{u}}{\sum_{u=1}^{n}\left({TB}_{u}+{FQ}_{u}\right)}. \end{array}$$

Therefore, the evaluation of the classifier by the two algorithms may be completely different.

## 4. Experimental Results of Teaching Mode of Basic Piano Course in Various Schools Based on Application Ability

Currently, a variety of schools have adopted the FC teaching method. The use of FC teaching mode is preferred by teachers and students in various schools for the instruction of basic piano courses, and it produces positive results. The FC teaching mode is still in its early stages, though. In order to analyze the FC, this paper uses the survey research methodology.

### 4.1. The Popularity of FC and the Help of FC to Teaching

In order to have a clearer understanding of the popularity of FC in various schools and the help of FC to basic piano courses in various schools, a random survey of 500 students in a music college is now conducted. Among them, the degree of understanding is divided into very understanding, general understanding, heard about it, and no understanding. Help situations are categorized as very helpful, generally helpful, may helpful, and not helpful, as shown in Figure 5.

As can be seen from Figure 5, the current level of college students' understanding of the FC is still relatively high, reaching 461. Most of the number of people focused on general knowledge and heard of it. There were only 39 people who did not know, and some students had little knowledge. In terms of help, because some students do not have a high degree of understanding of the FC teaching mode, a large number of students think that FC is helpful or may be helpful to basic piano lessons in various schools.

### 4.2. College Students' Recognition of the FC Teaching Model

In order to more objectively and comprehensively understand the practical effect of FC in basic piano courses in various schools, a random survey of 500 people in a music schools was conducted. This article focuses on investigating their recognition of the implementation of the FC teaching model in the basic piano courses in various schools. Recognition is divided into very like, somewhat like, average, dislike, and very dislike, as shown in Figure 6.

From the bar chart in Figure 6, it can be clearly seen that more than 80% of the students like the FC teaching mode, and only 2.8% of the students do not like this teaching mode. This data shows that students generally prefer the FC learning mode, which reflects the feasibility of using the FC teaching mode in college piano basic courses.

### 4.3. Comparison between Different Teaching Methods

The society's demand for applied piano talents determines the training direction of the applied piano education model, that is, to cultivate innovative talents and compound management talents. In the FC of basic piano courses in various schools, students are required to actively understand the required knowledge before class and learn in advance by consulting books, retrieving materials, and communicating with classmates. Based on this, the practical application ability of piano for college students is cultivated, so as to develop in an all-round way. Now, 500 students in various schools who participated in the FC are surveyed on “whether the FC is more conducive to the cultivation of application ability compared with the traditional classroom,” as shown in Figure 7.

In response to the question, “Compared with the traditional classroom, is the FC more conducive to the cultivation of application ability?” 80% of the students said that they thought the FC teaching mode was more effective at fostering application ability. This is more interesting and better suited for the development of practical talents than the traditional single teaching method used in many schools' basic piano courses. But 6% of the students still think that the FC is less effective than the conventional teaching methods at developing applied talents. This demonstrates that basic piano instruction, which is based on students' application skills in various schools, is still being delivered in an immature manner.

### 4.4. Comparison between Different Classes

In contrast to the conventional piano teaching method, the FC calls for students to hear the instructor explain things before class, come to their own conclusions, and then proceed with independent learning. Students have more opportunities to interact with teachers during set class times, and they can more effectively ask their own questions and clear up any confusions. Students can use instructional videos to practice the piano after class. A positive learning environment further encourages the growth of students' application ability. This method effectively increases students' participation in class and increases their enthusiasm for learning. The participation rate and enthusiasm of students under the traditional teaching mode and the FC were compared, and the test period was one year, in order to compare how well the two teaching methods cultivated students' application skills. The details are shown in Figure 8.

Figure 8 examines the comparison of student participation and motivation in learning in traditional and FC. Overall, it can be seen that the classroom participation rate and enthusiasm in the FC teaching mode are significantly higher than those in the traditional classroom teaching mode. From the perspective of classroom participation rate, there are fluctuations in both teaching modes, but the classroom participation rate under the FC teaching mode obviously increases steadily.

### 4.5. Comparison of the Training Situation in Different Classrooms

In piano teaching, the combination of theory and practice is required. In order to compare the cultivation of different classrooms, the current research investigates the cultivation of students' application ability in traditional classrooms and FC, as shown in Figure 9.

Figure 9 shows that in the flipped classroom teaching mode, students' application ability is significantly higher than in the traditional teaching mode. Students in the FC demonstrated an upward trend in their application ability, which grew steadily until it reached 75 points.

### 4.6. Comparison of Employment Rates in Different Classrooms

The ultimate purpose of using flipped classroom teaching is to improve the employment rate of students, and application ability is the key to improving the employment rate of students. A survey of the employment rate of graduates who use the FC teaching mode and the traditional teaching mode in a music college is now conducted. The survey period is from 2018 to 2022, and the specific situation is shown in Figure 10.

As can be seen from Figure 10, the annual employment rate under the FC teaching model is significantly higher than that of the traditional teaching model. The employment rate under the traditional teaching mode is up to 75%, and the employment rate under the FC teaching mode is up to 89%. Overall, the employment rate under the FC teaching mode is higher than that under the traditional teaching mode, and the employment rate has increased by an average of 14.2% and a maximum increase of 17%. This shows that the flipped classroom teaching mode is relatively successful for the basic piano course teaching mode in various schools based on students' application ability.

## 5. Conclusion

Major various schools are implementing educational reforms in order to cultivate piano talents as piano education has become more widely accepted. It actively develops students' application skills while enhancing students' musical literacy. The development of different schools to cultivate students' application ability is determined by the demand for application-oriented piano talents in society. As a result, the FC teaching mode is employed in various schools' basic piano courses in order to develop students' application skills. The FC teaching method is undoubtedly more well-liked by students than the conventional teaching method and can increase students' interest in learning. It significantly increases students' engagement and enthusiasm in class, develops their ability to apply knowledge, and supports the growth of their all-around competence. The way that basic piano lessons are taught in different schools is greatly impacted by the changes in society. The primary issue of the lack of applied talents in various schools can be resolved with the application of the FC teaching mode to the teaching of basic piano courses in various schools, which will also help to meet the demand for applied piano talents in the current society.

## Figures and Tables

**Figure 1:** Application-oriented college ternary interaction.

**Figure 2:** The difference between FC and traditional teaching.

**Figure 3:** Flipped classroom teaching mode.

**Figure 4:** Circular FC four-stage model.

**Figure 5:** The popularity of FC in colleges and universities and the help of FC to basic piano courses in colleges and universities.

**Figure 6:** Practical recognition of the implementation of FC teaching mode in basic piano courses in colleges and universities.

**Figure 7:** Compared with traditional classroom teaching, whether FC is more conducive to the cultivation of application ability.

**Figure 8:** Comparison of classroom participation rate and enthusiasm in traditional classroom and FC teaching mode.

**Figure 9:** The cultivation of students' application ability under the traditional classroom and FC teaching mode.

**Figure 10:** Comparison of the employment rate of college students under the traditional classroom and FC teaching mode.

## Data Availability

The data used to support the findings of this study are available from the corresponding author upon request.
